# Influence of Optimal Management of Hyperglycemia and Intensive Nursing on Blood Glucose Control Level and Complications in Patients with Postoperative Cerebral Hemorrhage

This article has been retracted.

**DOI:** 10.1155/2022/8553539

**Published:** 2022-08-29

**Authors:** Dandan Sun, Liang Sun, Fang Su

**Affiliations:** Neurosurgery, The First Affiliated Hospital of Soochow University, Suzhou 215006, China

## Abstract

**Background:**

Cerebral hemorrhage, also known as hemorrhagic stroke, is a common clinical cerebrovascular disease, accounting for about 10%-30% of stroke, with high morbidity and mortality.

**Objective:**

To observe the effect of optimal management of hyperglycemia and intensive nursing on blood glucose control level and complications in patients with postoperative cerebral hemorrhage.

**Methods:**

One hundred and eight patients with postoperative cerebral hemorrhage comorbid with stress hyperglycemia admitted to our neurosurgery department from February 2019 to February 2022 were selected and divided into a general group of 54 cases and an optimized group of 54 cases by simple random method. The general group was managed with conventional care, while the optimized group developed optimized management of hyperglycemia for intensive care. The indexes related to blood glucose control, electrolytes, National Institutes of Health Stroke Scale (NIHSS) scores, Barthel Index (BI) scores, and time to achieve blood glucose standard, insulin pumping time, patient satisfaction, and prognosis were compared between the two groups.

**Results:**

Before intervention, there was no statistical significance in the comparison of blood glucose control-related indicators and electrolytes between the two groups (*P* > 0.05). After 7 d and 14 d of intervention, the fasting blood glucose and 2 h postprandial blood glucose in the two groups were lower than before, while K+ and Na+ were higher than before (*P* < 0.05). The blood glucose indexes at the same time point in the optimized group were found to be lower than those in the general group by statistical analysis, but electrolytes were not statistically significant when compared with the general group (*P* > 0.05). In the optimized group, the time to achieve blood glucose standard (6.59 ± 1.94) d and insulin pumping time (7.14 ± 1.89) d were shorter than those in the general group [(7.48 ± 2.12) d and (8.58 ± 2.14) d], insulin dosage (748.85 ± 63.61) U was less than that in the general group (923.54 ± 84.14) U, and the incidence of hypoglycemia (3.70%) was lower than that in the general group (16.67%), and the satisfaction rate (92.59%) was higher than that of the general group (77.78%), which was statistically significant (*P* < 0.05). Before intervention, there was no significant difference in NIHSS score and BI score between the two groups (*P* > 0.05). After 7 d and 14 d of intervention, the NIHSS scores of the two groups were lower than before, while the BI scores were higher than before, and the NIHSS scores of the optimized group at the same time point were all lower than those of the general group, and the BI scores were higher than those of the general group (*P* < 0.05). The incidence of pulmonary infection (11.11%) and rebleeding (7.41%) in the optimized group were lower than those in the general group (25.93% and 22.22%), while deep vein thrombosis, multiple organ dysfunction syndrome (MODS), and death within 28 d was not statistically significant when compared with the general group (*P* > 0.05).

**Conclusion:**

Optimal management of hyperglycemia and intensive nursing can effectively control the blood sugar level of patients after cerebral hemorrhage, reducing insulin dosage, and the occurrence of hypoglycemia, pulmonary infection, and rebleeding.

## 1. Introduction

The formation of hematoma causes local brain tissue compression and ischemia, requiring surgical removal of the hematoma [1, 2]. Cerebral hemorrhage and surgery can cause stress response, with stress hyperglycemia as one of the main manifestations of stress hyperglycemia, but its mechanism is still unclear. Previous studies have shown that the disorder of neuroendocrine-humoral regulation system, abnormal secretion of various antiregulatory hormones, and disorder of blood glucose regulation-related hormones are one of the important mechanisms of stress hyperglycemia [3, 4].

It has been found that the incidence of stress hyperglycemia after cerebral hemorrhage is more than 50%, which is not only related to the severity of cerebral hemorrhage but also one of the independent risk factors affecting the neurological deficit and prognosis of patients with cerebral hemorrhage [5, 6]. At present, insulin is often used in clinical treatment of stress hyperglycemia, but there are still some patients with poor blood glucose control and many complications [7, 8]. Hyperglycemia optimal management intensive care is a care model focusing on glycemic control. This study observed the effect of hyperglycemia optimal management intensive care on the level of glycemic control and complications in postoperative patients with cerebral hemorrhage, which is reported below.

Core tips: stress hyperglycemia after cerebral hemorrhage is harmful, and effective control of blood glucose is the focus of postoperative treatment. In this study, patients with cerebral hemorrhage were treated with high blood glucose optimization management intensive nursing intervention. It was found that it can effectively control the blood glucose level of patients after cerebral hemorrhage, reduce the amount of insulin, and reduce the incidence of hypoglycemia, pulmonary infection, and rebleeding.

### 1.1. Data and Methods

#### 1.1.1. Case Selection

Inclusion criteria: (1) the cerebral hemorrhage met the criteria of the Chinese Guidelines for the Diagnosis and Treatment of Cerebral Hemorrhage [9], and the location of the hemorrhage was confirmed by brain CT; (2) the age was 18-75 years old, regardless of gender; (3) all patients were treated with minimally invasive surgery; (4) two consecutive random blood glucose values > 11.1 mmol/L and normal glycosylated hemoglobin (HbA1c); (5) the blood glucose was controlled by insulin pump; (6) no previous history of diabetes mellitus, and preoperative blood glucose levels were normal; (7) consent signed by the patient or his family.

Exclusion criteria: (1) history of drug use affecting blood glucose; (2) hyperglycemia due to diabetes and other diseases; (3) previous history of long-term glucocorticoid use; (4) presence of gastrointestinal damage, chronic constipation, and abnormal liver and kidney function; (5) poor overall condition of the patient with an expected survival of less than 6 months; (6) concomitant malignancy.

#### 1.1.2. Case Collection

One hundred and eight patients with postoperative cerebral hemorrhage comorbid with stress hyperglycemia admitted to our neurosurgery department from February 2019 to February 2022 were selected, of whom 58 were male and 50 were female; age ranged from 41 to 75 years, mean (61.89 ± 10.77) years, onset to admission time ranged from 3 h to 24 h, mean (7.89 ± 2.71) h. The simple randomization method was used to divide the patients into general group 54 cases and 54 cases in the optimized group, and the two groups of patients were comparable (*P* > 0.05).

### 1.2. Method

In the general group, conventional nursing management was adopted, and patients were instructed to eat low-salt, low-fat diet, quit smoking and alcohol, and were given comprehensive intervention such as reducing intracranial pressure, controlling blood pressure, blood lipids, antiplatelet, anticoagulation, nutritional nerve, and maintaining water and electrolyte balance. When the random blood glucose was >11.1 mmol/L, the continuous intravenous infusion of insulin was given. The blood glucose control objectives were fasting blood glucose < 6.1 mmol/L and postprandial 2 h blood glucose < 7.8 mmol/L.

The optimization group formulated hyperglycemia optimization management for intensive care. The intensive nursing intervention group was established to receive training on knowledge related to hyperglycemia optimization management, including the harm of stress hyperglycemia to the nervous system, the relationship between enteral nutrition and intravenous corresponding insulin dose, and hyperglycemia optimization management plan. The nursing staff performed all nursing operations according to the optimal hyperglycemia management plan, closely observed the condition, regularly monitored the blood glucose, and adjusted the nutrient intake and insulin dose according to the blood glucose monitoring results. If there is any abnormal blood glucose situation, it will be reported to the endocrinologist and neurosurgeon in time to give timely treatment. Insulin is administered by intravenous pump, and each insulin is administered for no more than 8 h. The nurse manager is responsible for monitoring the implementation of the program, including blood glucose monitoring, insulin dose adjustment, and data recording. Attention should be paid to identifying symptoms of hypoglycemia, especially in patients with disturbance of consciousness, such as sweating, rapid breathing, aggravation of disturbance of consciousness or blood glucose < 3.9 mmol/L immediately according to the hypoglycemic process, suspending insulin pumping, and quickly injecting 50% glucose injection.

### 1.3. Observation Indicators and Detection Methods

Blood glucose control-related indicators, electrolytes, National Institutes of Health Stroke Scale (NIHSS) score, Barthel index (BI) score, blood glucose compliance time, insulin pump time, patient satisfaction, and prognosis were compared between the two groups.

A total of 3 mL of venous blood specimens from the upper limbs of both groups were drawn before, 7 d and 14 d after the intervention, and fasting blood glucose and electrolyte indicators K+ and Na+ were measured by a fully automatic biochemical analyzer (Hitachi, model 7600, Japan). Blood was collected again 2 h after eating to test the postprandial 2 h blood glucose.

### 1.4. Score Standard

The satisfaction was measured by the hospital-made scale, including the environment, working ability of medical staff, and blood glucose control. The score was 0–100 points, and the score was proportional to the satisfaction. The score 90 or above was considered very satisfied, 70-90 was considered satisfied, and below 70 was considered dissatisfied. NIHSS score, with the range of 0-42 points, high or low score represented the size of nerve defect. BI score, with the range of 0-100 points, score level indicated the level of daily living ability.

### 1.5. Statistical Method

The data were processed by SPSS19.0. The K-S method was used to test the normality of measurement data such as age. The measurement data conforming to the normal distribution were described by (^−^*χ* ± *s*). The *t* test was used for comparison. The enumeration data such as gender were described by the number of cases (%). The *χ*^2^ test of four-grid table or row × list was used for comparison. *P* < 0.05 was statistically significant.

## 2. Results

### 2.1. Comparison of Baseline Data between Two Groups

There was no significant difference in the initial fasting blood glucose, body mass index, hematoma volume, admission GCS score, gender, age, smoking history, PT, Fib and PLT between the two groups (*P* > 0.05) (see Table 1).

### 2.2. Comparison of Blood Glucose Control between Two Groups

Before intervention, there was no significant difference in blood glucose control-related indicators between the two groups (*P* > 0.05). After 7 d and 14 d of intervention, the fasting blood glucose and 2 h postprandial blood glucose in the two groups were lower than those before intervention, and the blood glucose indexes at the same time point in the optimized group were statistically lower than those in the general group (*P* < 0.05) (see Table 2).

### 2.3. Comparison of Insulin Dosage and Blood Glucose Compliance Time between the Two Groups

The blood glucose compliance time and insulin pump time in the optimized group were shorter than those in the general group, the insulin dosage was less than that in the general group, and the incidence of hypoglycemia was lower than that in the general group, with statistical significance (*P* < 0.05) (see Table 3).

### 2.4. Comparison of Electrolyte between Two Groups

Before intervention, there was no significant difference in electrolyte between the two groups (*P* > 0.05). After 7 d and 14 d of intervention, K+ and Na+ in the two groups were higher than those before, but the electrolyte in the two groups at the same time was not statistically significant (*P* > 0.05) (see Table 4).

### 2.5. Comparison of Satisfaction between the Two Groups

The satisfaction of the optimized group was 92.59% (50/54), which was higher than 77.78% (42/54) of the general group, with statistical significance (*P* < 0.05) (see Table 5).

### 2.6. Comparison of NIHSS Score and BI Score between the Two Groups

Before intervention, there was no significant difference in NIHSS score and BI score between the two groups (*P* > 0.05). After 7 d and 14 d of intervention, the NIHSS score of the two groups decreased, while the BI score increased. The NIHSS score of the optimized group was lower than that of the general group at the same time point, and the BI score was higher than that of the general group (*P* < 0.05) (see Table 6).

### 2.7. Comparison of Prognosis between Two Groups

The incidence of pulmonary infection and rebleeding in the optimized group was lower than that in the general group, while the incidence of deep vein thrombosis, MODS, and death within 28 days in the optimized group was not statistically significant compared with that in the general group (*P* > 0.05) (see Table 7).

## 3. Discussion

Stress hyperglycemia is one of the common complications in neurocritical patients, and stress conditions can cause neuroendocrine disorders; as a result, stress hormones such as cortisol hormone, glucagon, and adrenal hormone are secreted in large amounts, promoting gluconeogenesis and causing massive hepatic glycogen synthesis. Neuroendocrine disorders can also lead to insulin resistance in the body [10–12]. Hematoma compression can lead to hypothalamus-pituitary-adrenal axis injury and reduce the biological uptake and utilization of glucose in peripheral tissues [13, 14]. In contrast, hyperglycemic state can affect brain tissue energy metabolism, leading to acidosis due to lactic acid accumulation and can induce oxidative stress, which aggravates neuronal cell damage and is detrimental to the prognosis of patients with cerebral hemorrhage [15, 16]. Therefore, clinical attention has been paid to the treatment of stress hyperglycemia in neurosurgical patients.

For patients with cerebral hemorrhage, dehydration to reduce intracranial pressure treatment can lead to blood viscosity, and the body is in a state of high catabolism after operation, which requires nutritional support treatment, and it is also easy to induce hyperglycemia [17, 18]. At present, the overall control effect of clinical stress hyperglycemia is not ideal. The reason for the poor therapeutic effect of insulin is not the problem of hyperglycemia, but the damage caused by large-scale blood glucose fluctuations and hypoglycemia [19, 20]. In this study, it was found that the fasting blood glucose and postprandial 2 h blood glucose of patients receiving intensive nursing intervention with optimized management of hyperglycemia after 7 d and 14 d were lower than those of patients receiving ordinary nursing intervention. The time of blood glucose reaching the standard and the time of insulin pump were shorter than those who received ordinary care intervention, the insulin dosage was less than those who received ordinary care intervention, and the incidence of hypoglycemia was lower than those who received ordinary care intervention. The above results suggest that intensive care for optimal management of hyperglycemia can effectively control the blood glucose level, reduce insulin dosage, and decrease hypoglycemia in patients after cerebral hemorrhage. This is due to high blood sugar optimization management intensive nursing intervention through regular monitoring of blood sugar, timely upload data to neurology and nutrition doctors, and jointly develop reasonable blood sugar control objectives, intervention of individualized insulin therapy, and nutritional intervention [21–23]. When insulin was injected intravenously, physiological insulin secretion mode was simulated as much as possible, and timely adjustment of enteral nutrition was helpful to control blood glucose fluctuation, effectively reduce blood glucose variability, and maintain blood glucose stability [24–26]. In this study, the electrolyte level was also detected. After intervention, K ^+^ and Na^+^ in the two groups increased, but there was no significant difference between the two groups. Because both groups attach importance to maintaining water-electrolyte balance during treatment.

In this study, it was found that the NIHSS score of patients receiving intensive nursing intervention with optimized management of hyperglycemia after 7 d and 14 d was lower than that of patients receiving ordinary nursing intervention, while the BI score was higher than that of patients receiving ordinary nursing intervention. The results suggest that the intensive nursing of hyperglycemia optimization management can effectively improve the degree of nerve defect and the ability of daily living in patients with cerebral hemorrhage after operation. This is due to the optimal management of hyperglycemia intensive nursing intervention mode of patients with better blood glucose control can avoid hyperglycemia damage to neurons [27–29]. Hyperglycemia can increase the anaerobic metabolism of brain tissue, destroy mitochondria, produce a large number of free radicals, and increase the Ca2 + influx of nerve cells [30–32]. Hyperglycemia can also cause excessive release and accumulation of excitatory amino acids such as glutamate, causing neuronal damage [33, 34].

This study also found that the incidence of pulmonary infection and rebleeding in patients receiving intensive nursing intervention with optimized management of hyperglycemia was lower than that in patients receiving ordinary nursing intervention, while there was no significant difference in the incidence of deep vein thrombosis, MODS, and death within 28 days between the two groups. Those who received intensive nursing intervention for optimal management of hyperglycemia were more satisfied than those who received ordinary nursing intervention. The above results suggest that intensive nursing of high blood glucose optimization management can reduce the risk of pulmonary infection and rebleeding. This is related to the improvement of immune function after stable blood glucose control, and stable blood glucose also helps to protect vascular endothelial cells and blood-brain barrier and prevent secondary brain injury and rebleeding [35].

In conclusion, intensive care for optimal management of hyperglycemia can effectively control the blood glucose level of patients after cerebral hemorrhage, reducing insulin dosage, and decreasing the occurrence of hypoglycemia, pulmonary infection, and rebleeding.

## Figures and Tables

**Table 1:** Comparison of baseline data between the two groups.

Normal information	General group (*n* = 54)	Optimized group (*n* = 54)	*χ* ^2^/*t*	*P*
Gender [*n* (%)]				
Male	30 (55.56)	28 (51.85)	0.149	0.700
Female	24 (44.44)	26 (48.15)		
Age [(^−^*χ* ± *s*), age]	61.74 ± 11.05	60.49 ± 11.41	0.578	0.564
Body mass index [(^−^*χ* ± *s*), kg/m^2^]	7.45 ± 2.86	7.91 ± 2.94	0.824	0.412
Initial fasting blood glucose [(^−^*χ* ± *s*), mmol/L]	9.57 ± 1.45	9.74 ± 1.29	0.644	0.521
Admission GCS score [*n* (%)]				
9-12 minutes	35 (64.81)	32 (59.26)	0.354	0.552
>12 minutes	19 (35.19)	22 (40.74)		
Hematoma volume [(^−^*χ* ± *s*), mL]	102.56 ± 35.89	99.74 ± 38.12	0.396	0.693
Smoking history [*n* (%)]				
Have	18 (33.33)	15 (27.78)	0.393	0.531
None	36 (66.67)	39 (72.22)		
PT [(^−^*χ* ± *s*), s]	18.52 ± 4.56	18.39 ± 4.74	0.145	0.885
Fib [(^−^*χ* ± *s*), g/L]	2.76 ± 1.02	2.71 ± 0.98	0.260	0.796
PLT [(^−^*χ* ± *s*), ×109/L]	231.56 ± 74.88	227.96 ± 81.04	0.240	0.811

**Table 2:** Comparison of blood sugar control between the two groups [(^−^*χ* ± *s*), mmol/L].

Group	*n*	Fasting blood sugar			2 h postprandial blood glucose		
		Before intervention	Intervention 7 d	Intervention 14 d	Before intervention	Intervention 7 d	Intervention 14 d
General group	54	9.57 ± 1.45	7.25 ± 1.23^∗^	5.75 ± 0.84^∗^	13.58 ± 3.85	10.05 ± 2.15^∗^	8.15 ± 1.36^∗^
Optimized group	54	9.74 ± 1.29	6.54 ± 1.04^∗^	5.23 ± 0.67^∗^	13.49 ± 3.79	8.56 ± 1.73^∗^	5.57 ± 1.04^∗^
*t*		0.644	3.239	3.556	0.122	3.968	11.074
*P*		0.521	0.002	0.001	0.903	0.000	0.000

Compared with before intervention, ^∗^*P* < 0.05.

**Table 3:** Comparison of insulin dosage and blood glucose reaching time between two groups.

Group	*n*	Blood sugar target time [(^−^*χ* ± *s*)*x*, d]	Insulin pump time [(^−^*χ* ± *s*), d]	Insulin dosage [(^−^*χ* ± *s*), U]	Hypoglycemia [*n* (%)]
General group	54	7.48 ± 2.12	8.58 ± 2.14	923.54 ± 84.14	9(16.67)
Optimized group	54	6.59 ± 1.94	7.14 ± 1.89	748.85 ± 63.61	2(3.70)
*χ* ^2^/*t*		2.276	3.706	12.170	4.960
*P*		0.025	0.000	0.000	0.026

**Table 4:** Comparison of electrolytes between the two groups [(^−^*χ* ± *s*), mmol/L].

Group	*n*	K^+^			Na^+^		
		Before intervention	Intervention 7 d	Intervention 14 d	Before intervention	Intervention 7 d	Intervention 14 d
General group	54	3.81 ± 0.15	4.15 ± 0.19^∗^	4.23 ± 0.23^∗^	134.25 ± 4.15	142.15 ± 6.98^∗^	148.85 ± 6.11^∗^
Optimized group	54	3.79 ± 0.18	4.18 ± 0.17^∗^	4.25 ± 0.28^∗^	132.98 ± 5.84	143.02 ± 5.84^∗^	146.78 ± 8.54^∗^
*t*		0.627	0.865	0.406	1.303	0.702	1.449
*P*		0.532	0.389	0.686	0.196	0.484	0.150

Compared with before intervention, ^∗^*P* < 0.05.

**Table 5:** Comparison of compliance between the two groups [*n* (%)].

Group	*n*	Very satisfied	Satisfy	Dissatisfied	Satisfaction
General group	54	19 (35.19)	23 (42.59)	12 (22.22)	42 (77.78)
Optimized group	54	28 (51.85)	22 (40.74)	4 (7.41)	50 (92.59)
*χ* ^2^					4.696
*P*					0.030

**Table 6:** Comparison of NIHSS scores and BI scores between the two groups [(^−^*χ* ± *s*), minute].

Group	*n*	NIHSS score			BI score		
		Before intervention	Intervention 7 d	Intervention 14 d	Before intervention	Intervention 7 d	Intervention 14 d
General group	54	19.02 ± 4.74	16.52 ± 3.15^∗^	12.23 ± 2.56^∗^	48.52 ± 8.56	56.96 ± 7.45^∗^	67.14 ± 6.22^∗^
Optimized group	54	18.89 ± 4.58	14.49 ± 2.87^∗^	10.04 ± 2.18^∗^	47.63 ± 9.11	63.22 ± 6.57^∗^	76.86 ± 6.35^∗^
*t*		0.145	3.501	4.786	0.523	4.631	8.036
*P*		0.885	0.001	0.000	0.602	0.000	0.000

Compared with before intervention, ^∗^*P* < 0.05.

**Table 7:** Comparison of prognosis between the two groups [*n* (%)].

Group	*n*	Deep vein thrombosis	MODS	Lung infection	Rebleeding	Die within 28 days
General group	54	3 (5.56)	5 (9.26)	14 (25.93)	12 (22.22)	3 (5.56)
Optimized group	54	1 (1.85)	1 (1.85)	6 (11.11)	4 (7.41)	1 (1.85)
*χ* ^2^		1.039	2.824	3.927	4.696	1.039
*P*		0.308	0.093	0.048	0.030	0.308

## Data Availability

The labeled dataset used to support the findings of this study are available from the corresponding author upon request.
